# The Effect of TLR9, MyD88, and NF-*κ*B p65 in Systemic Lupus Erythematosus

**DOI:** 10.1155/2022/6830366

**Published:** 2022-06-13

**Authors:** Huanan Wang, Feng Guo, Min Wang, Tingting Wang, Shanzhi Wang, Yanni Huang, Feng Ye

**Affiliations:** ^1^Department of Rheumatology and Immunology, The First Affiliated Hospital of Hainan Medical University, Haikou City 570102, Hainan Province, China; ^2^Department of Nephrology, The First Affillated Hospital of Hainan Medical University, Haikou City 570102, Hainan Province, China; ^3^School of Tropical Medicine and Laboratory Medicine, Hainan Medical University, Haikou City 570102, Hainan Province, China

## Abstract

**Purpose:**

This study was conducted to characterize the expression level of peripheral blood toll-like receptors 9 (TLR9), nuclear factor kappa-B protein 65 (NF-*κ*B p65), and myeloid differentiation factor88 (MyD88) of active systemic lupus erythematosus (SLE) and analyse their clinical significance.

**Methods:**

The prospective cohort study enrolled 30 active SLE patients (SG1 group), 30 stable SLE patients (SG2 group), and 20 healthy individuals (RG group) in the First Affiliated Hospital of Hainan Medical University between January 2018 and June 2020. All SLE patients were treated with methylprednisolone tablets. Quantitative polymerase chain reaction (qPCR) was used to determine the levels of TLR9, MyD88, and NF-*κ*B p65 in the peripheral blood mononuclear cell (PBMC). ELISA was adopted for the determination of serum interleukin (IL-6) and tumor necrosis factor-*α* (TNF-*α*).

**Results:**

Patients in SG1 showed the highest mRNA levels of TLR9, MyD88, and NF-*κ*B p65, followed by SG2, and then RG. SG1 had the highest serum levels of IL-6 and TNF-*α*, followed by SG2 and RG. The level of TLR9 was positively correlated with the SLE disease activity index (SLEDAI) and negatively correlated with complement component 3 (C3) and complement component 4 (C4). MyD88 and NF-*κ*B p65 were positively correlated with SLEDAI.

**Conclusion:**

Compared with a healthy status, SLE induces an increase in TLR9, MyD88, NF-*κ*B p65, IL-6, and TNF-*α* levels, and the activation of the TLR9-MyD88-NF-*κ*B p65 signal path was associated with the pathogenesis of SLE.

## 1. Introduction

SLE is an autoimmune inflammatory connective tissue disease with a high prevalence in young women. Its etiology is poorly understood and is considered to be associated with genetic factors or environmental factors [1]. During SLE, T cells and B cells are overactivated to produce large amounts of autoantibodies, causing widespread inflammation and tissue damage in the affected organs [2]. Manifestations of active SLE mainly include chest tightness, shortness of breath, and dyspnea [3]. In recent years, research has reported that TLRs act as transmembrane receptors that sense invading pathogens and are involved in the development of SLE by activating signaling pathways that affect both intrinsic and adaptive immunity [4]. As a member of the TLRs family, TLR9 plays a role in defending against pathogen invasion, releasing specific inflammatory factors, and activating multiple downstream signals such as MyD88 for immune response and other functions [5]. NF-*κ*B, as a transcriptional regulator, interacts with promoters and enhancers to regulate the activation of multicytokines and immune cells and participates in immune responses [6]. NF-*κ*B p65, a member of the NF-*κ*B family, forms a complex with inhibitors of NF-*κ*B (I*κ*B) and is located in the cytoplasm in an inactive form. When activated, the phosphorylation is dissociated from I*κ*B and enters the nucleus, where it binds to important genes in the nucleus for the regulation of downstream factors [7]. TLR9/MyD88/NF-*κ*B p65 is a classic pathway of inflammatory response that is closely related to various inflammatory diseases in the human body and participates in the development of inflammatory reactions [8]. The TLR9/MyD88/NF-*κ*B signaling pathway is potentially similar in the regulation of different diseases and is, therefore, the pharmacological basis of most drugs to treat diseases by regulating the levels of cytokines, inflammatory factors, and chemokines [9]. Studies have shown that a variety of traditional Chinese medicine (TCM) components play a role through TLR9/MyD88/NF-*κ* pathway [10, 11].

In this study, the TLR9, MyD88, and NF-*κ*B p65 in peripheral blood of active SLE patients were determined, and their correlation with SLE immunological indicators and their clinical significance were analyzed to investigate the pathogenesis of SLE and provide a basis for the prevention and treatment of SLE.

## 2. Materials and Methods

### 2.1. Study Design

The prospective cohort study enrolled 30 active SLE patients (SG1 group), 30 stable SLE patients (SG2 group), and 20 healthy individuals (RG group) in our hospital between January 2018 and June 2020. This research was performed under the ratification of the Ethics Committee of the First Affiliated Hospital of Hainan Medical University (Approval no. HN883001), and all patients and physical examinees understood the content of this research and voluntarily participated in the research. Undersigned informed consent has been obtained from all participants.

### 2.2. Inclusive and Exclusive Criteria

#### 2.2.1. Inclusive Criteria

Patients aged 10–65 years, who met the diagnostic criteria of SLE [12], and with complete clinical data and high compliance were included.

#### 2.2.2. Exclusion Criteria

Patients with RA, ankylosing spondylitis, and other immune diseases, with diabetes, infection, malignant tumor, and other diseases, and who were in pregnancy and lactation were excluded.

### 2.3. Treatment Methods

All patients with SLE received 1 mg/(kg·d) of prednisolone tablets (Approval number: H20020224, Tianjin Tianyao Medicine Pharmaceutical Co. Ltd.) for initial treatment, and the dose was reduced to 0.5 mg/(kg·d) after 8 weeks of treatment.

### 2.4. Clinical Outcome

#### 2.4.1. Blood Collection and Separation of Peripheral Blood Mononuclear Cell (PBMC)

5 ml of fasting venous blood was collected from all the participants, added with 5 ml of cell separation fluids, and centrifuged at 2000 rpm for 20 min to generate four liquid layers of the solution. The liquid of the thin PBMC band was collected, transferred to a new tube, and added with 12 ml of cell washing liquid, followed by centrifugation at 1500 rpm for 10 min. PBMCs were collected in the pellets at the bottom of the tubes.

#### 2.4.2. Real-Time Fluorescence Quantitative PCR

The total PBMC RNA was extracted via Trizol, and the cDNA was synthesized via a reverse transcription kit from Seymour Field. The reaction conditions were as follows: 37°C, 10 min; 90°C, 5 s. TLR9, MyD88, NF-*κ*B p65, and *β*-actin were amplified using a PCR instrument (WEALTEC). The primers were synthesized via Beijing Ambic Biotechnology Co., Ltd. The primer sequences and product lengths are shown in Table 1.

#### 2.4.3. ELISA of IL-6 and TNF-*α*

The protein IL-6 and TNF-*α* in serum were determined via ELISA kit (Nanjing Jisihuiyuan Biotechnology Co. Ltd.), and the sensitivity of the YT-MB96S microplate reader (Shandong Yuntang Intelligent Technology Co. Ltd.) was 100 *μ*g/L. The absorbance (*A* value) was determined at 450 nm in strict accordance with the instructions.

#### 2.4.4. SLE Activity Score (SLEDAI)

Patients in OG and SG2 were evaluated for mental symptoms, arthritis, facial erythema, neurological symptoms, oral ulcer, hair loss, blood vessels, inflammatory skin rash, and sensitivity to light. Moreover, routine blood and urine tests, complement component 3 (C3) and complement component 4 (C4), 24 h urinary protein, heart color ultrasonic diagnosis, chest CT, and anti-dsDNA indicators were performed and documented according to the standard SLEDAI scores.

### 2.5. Statistical Method

Statistical analysis was carried out using the SPSS19.0 software. The measurement data are expressed as (mean ± standard deviation) and analyzed using the *t*-test. Spearman analysis was performed for correlation analyses. Statistically significant results were defined as *P* < 0.05.

## 3. Results

### 3.1. General Data

In SG1, there were 5 males and 25 females, with a mean age of 37.43 ± 5.37 years, and a course of disease of 5.6 ± 2.1 years. In SG2, there were 6 males and 24 females, with a mean age of 36.86 ± 5.15 years and a course of disease of 5.7 ± 2.3 years. In RG, there were 3 males and 17 females with a mean age of 37.53 ± 5.57 years. There were no statistically significant differences in baseline information such as age and gender between the three groups (*P* > 0.05) (Table 2).

### 3.2. mRNA Expression Levels of TLR9, MyD88, and NF-*κ*B p65

The SG1 group showed the highest mRNA levels of TLR9, MyD88, and NF-*κ*B p65 in PBMC, followed by SG2 and RG (*P* < 0.05), as shown in Figure 1.

### 3.3. Serum Levels of IL-6 and TNF-*α*

The SG1 group showed the highest expression levels of IL-6 and TNF-*α*, followed by SG2, and then RG (*P* < 0.05), as shown in Figure 2.

### 3.4. Correlation Analysis

The level of TLR9 was positively correlated with the SLE disease activity index (SLEDAI) and negatively correlated with C3 and C4. MyD88 and NF-*κ*B p65 were positively correlated with SLEDAI, as shown in Table 3.

## 4. Discussion

SLE is mainly caused by cellular humoral immune disorders, and its deterioration may lead to multiorgan failure or even death. Therefore, investigation of the pathogenesis of SLE is the focus of clinical prevention and treatment of SLE [13].

TLRs are pattern recognition receptors (PRRs) that recognize early invading pathogens and activate innate immunity, playing a vital role in natural immunity and acquired immunity. As a member of the TLR family, TLR9 specifically recognizes bacterial and viral DNA and activates corresponding immune cells. Research has found that TLR9 transfers MyD88 from the cytoplasm to the endoplasmic reticulum through interaction with CpG DNA and interacts with the C-terminal TIR structure of MyD88 to activate MyD88, induce the release of inflammatory cytokines, and participate in the immune regulation [14]. MyD88 activates NF-*κ*B via signal molecules such as TAK1 and TRAF6. NF-*κ*B is a dimer-based transcriptional regulator that plays a key role in immune responses. NF-*κ*B p65 is a member of the NF-*κ*B family and regulates the release of IL-6 and TNF-*α* [15].

In the present study, it was found that active SLE was associated with the highest TLR9 levels in PBMC, followed by stable SLE, and a healthy status (*P* < 0.05). Previous research has reported a higher TLR9 level in SLE patients compared with the healthy population, suggesting the correlation of the TLR9 signaling pathway with the pathogenesis of SLE [5]. An animal study has found that lupus mice with TLR9 gene knockout showed significantly fewer lupus symptoms than lupus mice without TLR9 gene knockout [5], which also indicates a correlation between TLR9 and the pathogenesis of SLE. Research has also found that pathogen invasion and infection activate the upstream TLR9-MyD88-NF*κ*-B p65 signal path and induce the release of inflammatory cytokines and enzymes, leading to a cascade inflammatory reaction, which is associated with the pathogenesis of SLE [16, 17]. Moreover, it has been reported that TLR9 could induce the release of inflammatory cytokines by activating IL-1, NF-*κ*B, and other pathways [18]. Here, active SLE patients showed the highest levels of MyD88 and NF-*κ*B p65 in PBMC, followed by stable SLE patients, and then healthy participants (*P* < 0.05), suggesting a correlation between TLR9-MyD88-NF-*κ*B p65 signal path and SLE.

In addition, it was found in this study that SG1 had the highest levels of serum IL-6 and TNF-*α*, followed by SG2, and then RG (*P* < 0.05). TNF-*α* is involved in the pathogenesis of autoimmune diseases by inhibiting T cell signal transduction, promoting the growth of B cells and dendritic cells, and inducing the production of apoptotic molecules. Research has revealed a key role of TNF-*α* in the pathogenesis of SLE after obtaining significantly higher levels of TNF-*α* in SLE patients than those in healthy subjects [19]. In addition, TNF-*α* levels in stable SLE patients are higher than those in active SLE patients, suggesting that TNF-*α* may also be a protective cytokine for SLE [20]. IL-6 is an important Th2 cytokine involved in T and B lymphocyte-mediated inflammatory responses [21], and it has been shown in prior research that the serum IL-6 level in SLE patients is higher than that in healthy individuals, which is significantly positively correlated with SLEDAI and consistent with the results of the present study [22].

Furthermore, TLR9 expression levels were positively correlated with SLEDAI (*P* > 0.05) and negatively correlated with C3/C4 (*P* > 0.05), but not correlated with dsDNA (*P* > 0.05). MyD88 and NF-*κ*B p65 were positively correlated with SLEDAI (*P* > 0.05) but not with C3/C4 or dsDNA (*P* > 0.05). These results revealed that the signaling molecules in the TLR9-MyD88-NF-*κ*B p65 path are positively correlated with the SLEDAI and played different roles in the pathogenesis of SLE. Moreover, in addition to the C3/C4 and dsDNA, there were other factors involved in SLE activity. Studies have shown that the levels of TLR9, TGF-*β*1, and PDGF-B in peripheral blood of SLE patients are higher than those of normal controls, and patients with significantly increased TLR9 mRNA at the time of initial diagnosis may experience a poor prognosis in the short term, suggesting that TLR9 may be associated with the prognosis of SLE [23]. Studies have analyzed the levels of TLR9 and NF-*κ*B in peripheral blood mononuclear cells of SLE patients and found that the TLR9 level of SLE patients was significantly lower than that of normal controls, while the NF-*κ*B level was significantly higher [24]. There were several limitations in this study. It is a prospective cohort study with a limited sample size, and the results are susceptible to individual differences, which reduced the credibility. In addition, this study is not a prospective randomized control study, and there are deficiencies in the study design.

## 5. Conclusion

The TLR9, MyD88, NF-*κ*B, IL-6, and TNF-*α* were significantly upregulated in SLE patients. The TLR9-MyD88-NF-*κ*B p65 signal path was activated in SLE patients, which is associated with the pathogenesis of SLE. The signal molecules in this pathway played different roles in the pathogenesis of SLE, suggesting that proper intervention of these signaling molecules may potentially serve as the target for the prevention or treatment of SLE.

## Figures and Tables

**Figure 1:** mRNA expression levels of TLR9, MyD88, and NF-*κ*B p65. (a) mRNA expression levels of TLR9; (b) mRNA expression levels of MyD88; (c) mRNA expression levels of NF-*κ*B p65. ^*∗∗∗*^*P* < 0.001.

**Figure 2:** Serum levels of IL-6 and TNF-*α*. (a) Serum levels of IL-6. (b) Serum levels of TNF-*α*. ^*∗∗∗*^*P* < 0.001.

**Table 1:** Primer sequences.

	Forward primer	Reverse primer
TLR9	5′-GGGACCTCGAGTGTGAAGCA-3′	5′-CTGGAGCTCACAGGGTAGGAA-3′
MyD88	5′-GCACATGGGCACATACAC-3	5′-TGGGTCCTTTCCAGAGTTTG-3′
NF-*κ*B p65	5′-CTGAACCAGGGCATACCTGT-3′	5′-GAGAAGTCCATGTCCGCAAT-3′
*β*-Actin	5′-GGAGGGGCCGGACTCATC-3′	5′-CTCTATGCCAACACAGT-3′

**Table 2:** General data.

	Gender (male/female)	Age (years)	Disease course (years)
SG1 group	5/25	37.43 ± 5.37	5.63 ± 2.11
SG2 group	6/24	36.86 ± 5.15	5.74 ± 2.35
RG group	3/17	37.53 ± 5.57	NA
*χ*2/F/t	0.231	0.125	0.191
*P* value	0.891	0.833	0.849

**Table 3:** Correlation analysis of TLR9, MyD88, and NF-*κ*B p65 mRNA expression levels with experimental indicators.

Indicators	TLR9		MyD88		NF-*κ*B p65	
	*r*	*P* value	*r*	*P* value	*r*	*P* value
SLEDAI	0.895	<0.05	0.452	<0.05	0.535	<0.05
C3	−0.624	<0.05	−0.053	>0.05	−0.043	>0.05
C4	−0.646	<0.05	−0.065	>0.05	−0.032	>0.05
dsDNA	0.544	<0.05	0.013	>0.05	0.008	>0.05

## Data Availability

The datasets used during the present study are available from the corresponding author upon reasonable request.

## Abbreviations

TLR9: Toll-like receptor 9
NF-*κ*B: Nuclear factor kappa-B
MyD88: Myeloid differentiation factor 88
SLE: Systemic lupus erythematosus
SG1: Study group 1
SG2: Stable group 2
RG: Reference group
CG: Control group
OG: Observation group
PBMCs: Peripheral blood mononuclear cells
TLRs: Toll-like receptors
RA: Rheumatoid arthritis
PRR: Pattern recognition receptor.

## References

[1] Mu Q., Zhang H., Luo X. M. (2015). SLE: another autoimmune disorder influenced by microbes and diet?. *Frontiers in Immunology*.

[2] Hamilton J. A., Hsu H. C., Mountz J. D. (2019). Autoreactive B cells in SLE, villains or innocent bystanders?. *Immunological Reviews*.

[3] Weinstein A., Alexander R. V., Zack D. J. (2021). A review of complement activation in SLE. *Current Rheumatology Reports*.

[4] Fillatreau S., Manfroi B., Dörner T. (2021). Toll-like receptor signalling in B cells during systemic lupus erythematosus. *Nature Reviews Rheumatology*.

[5] Tilstra J. S., John S., Gordon R. A. (2020). B cell-intrinsic TLR9 expression is protective in murine lupus. *Journal of Clinical Investigation*.

[6] Kunnumakkara A. B., Shabnam B., Girisa S. (2020). Inflammation, NF-*κ*B, and chronic diseases: how are they linked?. *Critical Reviews in Immunology*.

[7] Białas N., Müller E. K., Epple M., Hilger I. (2021). Silica-coated calcium phosphate nanoparticles for gene silencing of NF-*κ*B p65 by siRNA and their impact on cellular players of inflammation. *Biomaterials*.

[8] Valovka T., Hottiger M. O. (2011). p65 controls NF-*κ*B activity by regulating cellular localization of I*κ*B*β*. *Biochemical Journal*.

[9] Jing R., Hu Z.-K., Lin F. (2020). Mitophagy-mediated mtDNA release aggravates stretching-induced inflammation and lung epithelial cell injury via the TLR9/MyD88/NF-*κ*B pathway. *Frontiers in Cell and Developmental Biology*.

[10] Shi Y., Xu H., Xiao Y. (2020). Gegen qinlian decoction downregulates the TLR7 signalling pathway to control influenza A virus infection. *Biomedicine & Pharmacotherapy*.

[11] Li L., Zang H., Jiang Y. (2021). Acupuncture at back-shu and front-mu acupoints prevents gastric ulcer by regulating the TLR4/MyD88/NF-*κ*B signaling pathway. *Evidence-Based Complementary and Alternative Medicine*.

[12] Aringer M., Johnson S. R. (2020). Classifying and diagnosing systemic lupus erythematosus in the 21st century. *Rheumatology*.

[13] Pan L., Lu M. P., Wang J. H., Xu M., Yang S. R. (2020). Immunological pathogenesis and treatment of systemic lupus erythematosus. *World Journal of Pediatrics: WJP*.

[14] Ngo V. N., Young R. M., Schmitz R. (2011). Oncogenically active MYD88 mutations in human lymphoma. *Nature*.

[15] Cop N., Ebo D. G., Bridts C. H. (2018). Influence of IL-6, IL-33, and TNF-*α* on human mast cell activation: lessons from single cell analysis by flow cytometry. *Cytometry Part B: Clinical Cytometry*.

[16] Deguine J., Barton G. M. (2014). MyD88: a central player in innate immune signaling. *F1000Prime Reports*.

[17] Kim Y.-C., Lee S. E., Kim S. K. (2019). Toll-like receptor mediated inflammation requires FASN-dependent MYD88 palmitoylation. *Nature Chemical Biology*.

[18] Li Y., Liu M., Zuo Z. (2017). TLR9 regulates the NF-*κ*B-NLRP3-IL-1*β* pathway negatively in salmonella-induced nkg2d-mediated intestinal inflammation. *The Journal of Immunology*.

[19] Aringer M., Smolen J. S. (2012). Therapeutic blockade of TNF in patients with SLE-promising or crazy?. *Autoimmunity Reviews*.

[20] Postal M., Appenzeller S. (2011). The role of tumor necrosis factor-alpha (TNF-*α*) in the pathogenesis of systemic lupus erythematosus. *Cytokine*.

[21] Yao X., Huang J., Zhong H. (2014). Targeting interleukin-6 in inflammatory autoimmune diseases and cancers. *Pharmacology & Therapeutics*.

[22] Schubert C., Seizer L., Chamson E. (2021). Real-life cause-effect relations between urinary IL-6 levels and specific and nonspecific symptoms in a patient with mild SLE disease activity. *Frontiers in Immunology*.

[23] Yuan Y., Zhao L., Ye Z., Ma H., Wang X., Jiang Z. (2019). Association of toll‑like receptor 9 expression with prognosis of systemic lupus erythematosus. *Experimental and Therapeutic Medicine*.

[24] Li X.-L., Zhang Z., Zhang H. (2019). Expression level of TLR9, but not hypomethylation, is correlated with SLE disease activity. *Physiological Research*.

